The article "Polydatin improves osteogenic differentiation of human bone mesenchymal stem cells by stimulating TAZ expression via BMP2-Wnt/β-catenin signaling pathway" was retracted in 2023. Reasons: results that could not be reproduced; errors in the materials.

# Polydatin improves osteogenic differentiation of human bone mesenchymal stem cells by stimulating TAZ expression via BMP2-Wnt/β-catenin signaling pathway

**DOI:** 10.1186/s13287-020-01705-8

**Published:** 2020-05-27

**Authors:** Ying-Shan Shen, Xiao-Jun Chen, Sha-Na Wuri, Fan Yang, Feng-Xiang Pang, Liang-Liang Xu, Wei He, Qiu-Shi Wei

**Affiliations:** 1 First Clinical Medical College, Guangzhou University of Chinese Medicine, Guangzhou, Guangdong China; 2 Key Laboratory of Orthopaedics & Traumatology, The First Affiliated Hospital of Guangzhou University of Chinese Medicine, Guangzhou University of Chinese Medicine, Guangzhou, China; 3 Hip Preserving Ward, No. 3 Orthopaedic Region, The First Affiliated Hospital of Guangzhou University of Chinese Medicine, Guangzhou, Guangdong China; 4 No. 3 Orthopaedic Region and Institute of the Hip Joint, The First Affiliated Hospital of Guangzhou University of Chinese Medicine, Guangzhou, Guangdong China; 5 Third Clinical Medical College, Guangzhou University of Chinese Medicine, Guangzhou, Guangdong China; 6 The Third Affiliated Hospital of Guangzhou University of Chinese Medicine, Guangzhou, Guangdong China; 7 Institute of orthopedics of Guangzhou University of Chinese Medicine, Guangzhou, Guangdong China

**Keywords:** Polydatin, Human bone marrow stromal cells, Osteogenic differentiation, Transcriptional coactivator with PDZ-binding motif

## Abstract

**Objectives:**

Polydatin (PD), extracted from *Polygonum cuspidatum*, has shown potential therapeutic applications due to its antiosteoporotic and anti-inflammatory activities. Our previous study suggested that PD promotes the osteogenesis of human bone marrow stromal cells (hBMSCs) via the BMP2-Wnt/β-catenin pathway. The aim of our present study was to further explore the role of PD-mediated regulation of Tafazzin (TAZ), a transcriptional coactivator with a PDZ-binding motif, in osteogenesis.

**Materials and methods:**

hBMSCs were isolated and treated with PD at various concentrations. Alizarin red staining and RT-qPCR were performed to identify calcium complex deposition in hBMSCs as well as the expression of specific osteoblast-related markers, respectively, in each group. Next, TAZ-silenced hBMSCs were generated by lentivirus-produced TAZ shRNA. After treatment with PD, the osteogenic abilities of the TAZ-silenced and control hBMSCs were estimated by ALP activity assay, and expression of the TAZ protein was detected by Western blot analysis and immunofluorescence staining. In vitro, an ovariectomized (OVX) mouse model was established and used to evaluate the effect of PD on bone destruction by micro-CT, immunohistochemistry, and ELISA.

**Results:**

In vitro, 30 μM PD significantly improved the proliferation and calcium deposition of hBMSCs and markedly stimulated the expression of the mRNAs *RUNX2*, *Osteopontin*, *DLX5*, *β-catenin*, *TAZ*, and *Osteocalcin* (*OCN*). Osteogenic differentiation induced by PD was blocked by lentivirus-mediated TAZ shRNA. Furthermore, Noggin (a regulator of bone morphogenic protein 2 (BMP2)) and DKK1 (an inhibitor of the Wnt/β-catenin pathway) were found to inhibit the increase in TAZ expression induced by PD. In vivo, PD prevented estrogen deficiency-induced bone loss in the OVX mouse model.

**Conclusion:**

Taken together, our findings suggest that PD improved the osteogenic differentiation of hBMSCs and maintained the bone matrix in the OVX mouse model through the activation of TAZ, a potential target gene of the BMP2-Wnt/β-catenin pathway.

## Introduction

Osteoporosis (OP) is a bone metabolic disease characterized by reduced bone density and an increased risk of bone fracture [1, 2]. More than 20% of males and 50% of females older than 50 have experienced a decrease in bone density; thus, the annual medical expense for hip fracture in the USA is expected to rise to $67.7 billion by 2020 [3]. To date, the pathogenesis of OP is still unclear, but multiple important pathogenic factors, including age, sex, and steroid treatment, have been identified. Additionally, growing evidence indicates that defective osteogenic differentiation of bone marrow stromal cells (BMSCs) might lead to the occurrence of OP [4, 5]. Thus, promoting the osteogenesis of BMSCs may be a promising strategy for the treatment of OP.

In recent years, cell therapy has emerged as an effective approach for bone regeneration. BMSCs, the progenitor cells in skeletal tissues, play a critical role in cell differentiation in cell types such as osteoblasts, adipocytes, and chondrocytes [6, 7] through specific signaling pathways. The Wnt/β-catenin and BMP pathways have been shown to be essential in the osteogenic differentiation of BMSCs [4, 8]. When Wnt ligands bind the receptors LRP5/6 and Frizzled receptors, the classical Wnt/β-catenin pathway is activated, after which formation of the Wnt-fz-lrp6 complex (including Axin, APC, GSK3, and CK1) promotes the release of β-catenin [9–13]. Ultimately, β-catenin migrates to the nucleus, where it forms a complex with TCF/LEF to stimulate the expression of osteogenic genes, such as *RUNX2*, *ALP*, *DLX5*, and *OCN* [14, 15]. Wnt3a, a ligand of Wnt, has been proven to bind BMP proteins to activate a series of downstream reactions and promote osteogenic differentiation of BMSCs [16]. BMP2, one of the most important cytokines of the TGFβ1 superfamily [17], can promote the expression of Wnt3a and FZ and the activity of TCF/LEF and increase the expression of Wnt3a protein [18, 19]. Moreover, BMP2 has the capacity to stimulate osteogenic differentiation of BMSCs by increasing the expression and phosphorylation of β-catenin [15]. All these findings support the critical roles of the BMP2 and Wnt/β-catenin pathways and their crosstalk in inducing osteoblastic differentiation of BMSCs.

As a transcriptional coactivator in the Hippo signaling pathway, transcriptional coactivator with Tafazzin (TAZ) plays a regulatory role in the Wnt signaling pathway [20]. A previous study confirmed the functions of TAZ, such as its mediation of the osteogenic differentiation of adipose-derived stem cells [21]; remarkably, TAZ obviously accelerated the osteogenesis of BMSCs through increasing the expression of RUNX2, a key transcription factor in the BMP and Wnt/β-catenin pathways [22, 23]. All these findings indicate that TAZ serves as a vital osteogenesis mediator in BMSCs. In addition, our former study highlighted the pivotal role of TAZ in the osteogenic differentiation of BMSCs stimulated by the natural compound icariin via the estrogen receptor (Era) and Wnt/β-catenin signaling pathways [24].

Polydatin (PD), an important Chinese compound famous for its effects against inflammation, oxidation, and scar hyperplasia, can also improve the migration of BMSCs through the ERK 1/2 signaling pathway [25–29]. PD was recently found to alleviate osteoporosis symptoms in the ovariectomized (OVX) mouse model by upregulating the expression of β-catenin [30]. Previously, we showed the osteogenetic effect of PD on hBMSCs through the BMP-Wnt/β-catenin pathway [31].

In the present study, we aimed to investigate whether TAZ acts as a downstream transcriptional factor of the BMP2-Wnt/β-catenin pathways during the osteogenic differentiation of hBMSCs stimulated with PD. The inhibitory effect of PD altered the progression of OVX mice. Our results showed that PD promoted the proliferation and osteogenic differentiation of hBMSCs and prevented bone loss in the OVX mouse model. Moreover, TAZ played a critical role in this process, as supported by the effect of shTAZ, which reversed the effect of TAZ on osteogenesis. Therefore, TAZ may serve as a decisive factor involved in the osteogenic effect of PD in hBMSCs, as well as the antiosteoporosis effect of PD, through the BMP2-Wnt/β-catenin signaling pathway.

## Materials and methods

### Reagents and antibodies

hBMSCs were obtained from Cyagen Bioscience (Guangzhou, China). PD (purity ≥ 94%) was purchased from the National Institutes for Food and Drug Control (Beijing, China). Recombinant human Dickkopf-related protein 1 (DKK1) and Noggin were obtained from PeproTech (Rocky Hill, NJ, USA). Ficoll medium to generate a Ficoll density gradient was purchased from GE Healthcare (Silverwater, Australia). Fetal bovine serum (FBS), low-glucose Dulbecco minimum essential medium (LG-DMEM), and penicillin-streptomycin were obtained from Gibco-BRL (Gaithersburg, MD, USA). An MTT assay kit, β-glycerophosphate, dexamethasone, dimethyl sulfoxide (DMSO), and l-ascorbic acid-2-phosphate were all purchased from Sigma (Steinheim, Germany). Alizarin red was obtained from Aladdin Company, and an alkaline phosphatase activity measurement kit was obtained from Nanjing Jiancheng Company (Nanjing, China). pLent-U6-GFP-Puro vector was obtained from GenePharma Company (China). SYBR® Premix Ex TaqTM II and Prime Script TM RT Master Mix were purchased from Takara Biotechnology Company (Dalian, China). Anti-β-catenin antibody, anti-β-actin antibody, secondary antibodies, and phosphor-β-catenin (p-β-catenin) were obtained from Santa Cruz (Paso Robles, CA, USA). Chemiluminescence reagents were purchased from Pierce (Rockford, IL, USA).

### Cell extraction and culture

hBMSCs were separated and expanded following a previously described method [32]. Briefly, the human bone marrow was isolated using a Ficoll density gradient. Then, suspended cells were seeded into culture flasks after washing the MSC-enriched fraction. All flasks were maintained in an incubator with a humidified atmosphere at 37 °C and 5% CO_2_, and the medium was replaced every 4 days. After reaching confluence, the cells were passaged to the third generation. hBMSC surface markers (CD44 and HLA-DR) were identified by flow cytometry. Third-generation hBMSCs were used in the following experiments.

Cells were treated with PD at four different concentrations (0, 10, 30, or 100 μM) in the presence of osteogenic induction medium (OIM) consisting of l-ascorbic acid-2-phosphate (50 mM), dexamethasone (10^−8^ mol/L), and β-glycerophosphate (10^−2^ mol/L) to determine the optimal concentration of PD to increase the proliferation and osteogenic differentiation of hBMSCs. The following four different groups of cells were set to ascertain the effects of PD, Noggin, and DKK1 on the osteogenic differentiation of hBMSCs: group 1, which was cultured with PBS and OIM; group 2, which was cultured with PD and OIM; group 3, which was cultured in a mixture of OIM, PD, and 10^−7^ M Noggin; and group 4, which was cultured in a mixture of OIM, PD, and 2 mg/mL DKK1 [33].

### Cell proliferation assay

The MTT assay was used to determine the effect of PD on the proliferation of hBMSCs. Cells (1 × 10^4^ per well) were plated in 96-well plates and maintained in basic medium for 24 h. When the hBMSCs were 80% confluent, they were starved for 12 h without serum and then incubated in OIM with or without PD at different concentrations (0, 30, 10, 100 μM) for 1, 2, 3, 7, and 14 days. In addition, hBMSCs were cultured in a medium containing MTT (5 mg/mL) for 3 h at each of these time points at 37 °C. After the formazan crystals had dissolved in DMSO, the absorbance at 570 nm was measured with a microplate reader (Thermo Scientific, Waltham, MA, USA).

### Alizarin red staining

hBMSCs were seeded into 24-well plates and cultured in OIM with PD at different doses (0, 30, 10, and 100 μM) at 37 °C and 5% CO_2_ for 21 days. Then, the cells were washed with PBS twice and fixed with 97% ethanol for 10 min. The hBMSCs were then washed three times with deionized water and stained with a 0.1% Alizarin red staining solution (pH 8.3) for 30 min at room temperature. After the Alizarin red solution was removed, the hBMSCs were rinsed with deionized water and PBS twice each and then dried at room temperature. The cells were observed using a 450 fluorescent inverted phase contrast microscope (Nikon Corporation, Tokyo, Japan).

### Real-time quantitative PCR analysis

Total RNA was extracted at predetermined time points (3, 7, and 14 days), including groups 1–4 and groups A–D, using the MAGNET Total RNA Kit using a Thermo Scientific KingFisher Duo system. The RNA concentration was determined by a microplate reader. cDNA templates were synthesized using a Takara Prime Script II 1st Strand cDNA Synthesis Kit (D6210A). Real-time quantitative PCR (qPCR) was carried out using SYBR® Premix Ex TaqTM in a thermocycler. The qPCR conditions were as follows: denaturation at 93 °C for 180 s, followed by 30 cycles of 94 °C for 30 s and 60 °C for 30 s. β-Actin was used as an internal reference in all analyses, and the 2ΔΔCt method was used to calculate the data. All analyses were carried out in triplicate. The primer sequences are shown in Table 1.

**Table 1:** The primer sequences used in the present study

Gene	Gene ID	Sequence (5′-3′)	Product length (bp)
TAZ	XM_006229600.2	Forward: ACCCGCGAGTACAACCTTCTT	173
		Reverse: TATCGTCATCCATGGCGAACT	
RUNX2	NM_001015051.3	Reverse: GGGTGGGTCTCTGTTTCAGG	112
		Reverse: GTAGTGACCTGCGGAGATTAAC	
Osteopotin	NM_000582.2	Forward: CATATGATGGCCGAGGTGATAG	108
		Reverse: AGGTGATGTCCTCGTCTGTA	
DLX5	NM_005221.5	Forward: CCAACCAGCCAGAGAAAGAA	113
		Reverse: TAATGCGGCCAGCTGAAA	
OCN	NM_199173.5	Forward: CTAAAGGCGAACCTGGTGAT	105
		Reverse: CAGCCTCCAGCACTGTTTAT	
β-Catenin	NM_001098209.1	Forward: CTTCACCTGACAGATCCAAGTC	98
		Reverse: CCTTCCATCCCTTCCTGTTTAG	
Collagen type I	NM_000088.3	Forward: CTAAAGGCGAACCTGGTGAT	107
		Forward: CTAAAGGCGAACCTGGTGAT	
BMP2	NM_001200.3	Forward: TGCTTCTTAGACGGACTGCG	243
		Reverse: GGGTGGGTCTCTGTTTCAGG	
OPG	NM_002546.3	Forward: ACGCGGTTGTGGGTGCGA	354
		Reverse: AAGACCGTGTGCGCCCCTTG	
GAPDH	NM_001256799.2	Forward: CAAGAGCACAAGAGGAAGAGAG	102
		Reverse: CTACATGGCAACTGTGAGGAG	

### Amplification and purification of lentivirus-mediated TAZ shRNA

Short hairpin RNA (shRNA) duplex targeting TAZ mRNA (shTAZ) was synthesized, and a nontargeting oligo duplex (shCON) served as a negative control. The pLent-U6-GFP-Puro vector was used to prepare the lentiviral vector (LV). shTAZ was cloned into the lentiviral vector according to the manufacturer’s protocol. The lentiviral vector (LvshTAZ), pHelper 1.0 plasmid, and pHelper 2.0 helper plasmid were cotransfected into HEK293T cells to prepare lentiviral particles. Viral supernatants were harvested at 48 h after transfection and applied to hBMSCs in α-MEM containing 10% FBS and 8 mg/mL polybrene. Cells were incubated for 24 h with 2 mg/mL puromycin to remove uninfected cells. After 1 week of selection, the cells were used in the differentiation experiment. TAZ levels were certified by Western blot analysis and qPCR. The following are the shTAZ and shCON sequences:

shTAZ#1: 5′-GATCCGCTTCTGGACCAAGTATATGAACTTCAAGAGAGTTCATATACTTGGTCCAGAAGCTTTTTTA-3′, 5′-CGCGTAAAAAAGCTTCTGGACCAAGTATATGAACTCTCTTGAAGTTCATATACTTGGTCCAGAAGC-3′

shTAZ#2: 5′-GATCCGCCACATCTGGAACCTGAAGTTGTTCAAGAGACAACTTCAGGTTCCAGATGTGGCTTTTTTA-3′, 5′-CGCGTAAAAAAGCCACATCTGGAACCTGAAGTTGTCTCTTGAACAACTTCAGGTTCCAGATGTGGC-3′

shTAZ#3: 5′-GATCCGGCAAATGTGTGCCTGTATGTCGTTCAAGAGACGACATACAGGCACACATTTGCCTTTTTTA-3′, 5′-CGCGTAAAAAAGGCAAATGTGTGCCTGTATGTCGTCTCTTGAACGACATACAGGCACACATTTGCC-3′

shCON: 5′-GATCCGCCTAAGGTTAAGTCGCCCTCGCTCGAGCGAGGGCGACTTAACCTTAGGTTTTTA-3′, 5′-CGCGTAAAAACCTAAGGTTAAGTCGCCCTCGCTCGAGCGAGGGCGACTTAACCTTAGG-3′

### ALP activity assay

hBMSCs were seeded into 48-well plates (2 × 10^4^ per well) and incubated at 37 °C and 5% CO_2_. After reaching 80% confluence, the cells were cultured in OIM without or with PD at different concentrations (10, 30, and 100 μM) for 1, 2, 3, 7, and 14 days. hBMSC lysates were subjected to ALP activity examination by a commercial ALP assay kit (Abcam, Cambridge, MA, USA).

### Western blot analysis

At the indicated time points (3, 7, and 14 days), hBMSCs were separately lysed with RIPA lysis buffer consisting of Tris-HCl (50 mM, pH 8.0), NaCl (150 mM), 1% NP-40, 0.5% sodium chloride, and 0.1% sodium dodecyl sulfate. The lysate protein concentration was measured with a Bradford protein assay kit. All samples were separated by 10% SDS-PAGE and electrotransferred to the PVDF membranes. The membranes were blocked with 5% fat-free milk and incubated overnight at 4 °C with the primary antibodies anti-TAZ, anti-pTAZ Ser89, and anti-β-actin. The membranes were incubated with secondary antibody for 1 h after rinsing with PBS containing Tween-20 three times. Immunoreaction signals were detected by an enhanced chemiluminescence detection kit, and the images were analyzed using the Quantity One software. Band intensity was quantified and normalized against β-actin.

### Immunofluorescence staining

After 14 days of treatment, hBMSCs (groups A–D) were fixed with cold acetone for 15 min at room temperature, permeabilized (0.25% Triton X-100 in PBS for 15 min), and then blocked in 0.1% Triton X for 20 min. To block nonspecific antibody binding, cells were incubated for 20 min with 1% bovine serum albumin (BSA) and then incubated with primary anti-β-catenin antibody (1:200) at 4 °C overnight. The next day, the cells were incubated with a 1:500 dilution of rabbit secondary antibody labeled with APC for 1 h. After the cells were rinsed with PBS, the nuclear translocation of β-catenin was visualized by staining with 4′-6-diamidino-2-phenylindole (DAPI). Stained hBMSCs were examined under a fluorescence microscope, and images were captured with the Image Manager software.

### OVX mouse model

All experiments were authorized by the Institutional Animal Ethics Committee of Guangzhou University of Chinese Medicine and performed under the guidelines set forth by the National Institutes of Health Guidelines for the Care and Use of Laboratory Animals. Eighteen 7-week-old specific pathogen-free C57BL/6J female mice were randomly divided into three groups: (1) sham group (served as controls without any treatment, *n* = 6), (2) OVX group (mice whose ovaries were removed, *n* = 6), and (3) OVX+PD group (ovariectomized mice treated with 3 mg/kg PD by intraperitoneal injection, *n* = 6). The mice underwent standard feeding in cages (three mice per cage) under a 12-h light/dark cycle. After anesthetization, mice in the OVX group and OVX+PD group underwent ovariectomy to induce estrogen deficiency, while mice in the sham group underwent ovariectomy in the same manner, except a small amount of fat tissue beside the ovaries was removed. Each ovary removed from mice in the OVX and OVX+PD groups was completely removed, including its capsule and part of the oviduct. Mice in all of the groups had 1 week for recovery and incision healing. After that, mice in the OVX+PD group were given an intraperitoneal injection of 3 mg/kg PD every 2 days, instead of the 1% DMSO administered to mice in the sham and OVX groups. After predetermined durations (4, 8, and 12 weeks), the femurs of the mice were removed after sacrifice for subsequent histological and micro-CT examinations. The serum was extracted from the abdominal aorta of the mice in every group, and the protein levels of osteoclastogenesis inhibitory factor (OPG), RANKL, OPG/RANKL, and β-CTX were evaluated using ELISA kits according to the manufacturers’ instructions.

### Micro-CT analysis

The femurs were fixed overnight in 10% neutral buffered formalin and analyzed by SkyScan 1176 micro-CT equipment (SkyScan, Aartselaar, Belgium). The scanner was set at a resolution of 9 μm per pixel. The proximal femur beginning at 0.5 mm above the bottom of the growth plate and extending for 1 mm was chosen as the region of interest (ROI) used to determine the trabecular thickness (Tb.Th), trabecular separation (Tb.Sp), bone volume per tissue volume (BV/TV), bone surface area per bone volume (BS/BV), structure model index (SMI), and trabecular number (Tb.N).

### Histological and immunohistochemical analyses

The samples were fixed in 4% paraformaldehyde (PFA) for 24 h and then decalcified. All samples were cut into 5-μm sections and stained using hematoxylin and eosin (H&E) for histological observation. The extent of osteogenesis was evaluated by immunohistochemical (IHC) analysis of TAZ and OCN. Images were acquired with the Aperio ScanScope (Leica Biosystem, Buffalo Grove, IL, USA), and bone histomorphometric analyses were performed using the BIOQUANT OSTEO software (Bioquant Image Analysis Corporation, Nashville, TN, USA).

### Statistical analysis

The results are shown as the mean ± standard deviation (SD). One-way ANOVA was used to analyze data from multiple groups using SPSS version 19.0 (SPSS, Inc., USA). A *p* value of less than 0.05 indicated statistical significance.

## Results

### Phenotype identification of hBMSCs

hBMSCs at passages 2 and 3 were 90% confluent after 3 days of culture (Fig. 1a). As shown in Fig. 1b, passage 2 cells were tested by flow cytometry. The results indicated that 94.4% of cells were positive for CD44, while 0.4% were negative for HLA-DR. Hence, the majority of the isolated and purified cells expressed markers characteristic of hBMSCs.

**Fig. 1:** Morphology (**a**) and identity (**b**) of human bone marrow stromal cells (hBMSCs). The hBMSCs were identified with CD44 (94.4%) and HLA-DR (0.4%) compared with the corresponding isotype control

### Polydatin promoted the proliferation and osteogenic differentiation of hBMSCs

hBMSCs were cultured in a basal medium with or without PD at various concentrations (10, 30, and 100 μM) for 1–14 days. The results of the MTT assay showed that 30 μM PD treatment significantly improved hBMSC proliferation at each time point (*p* < 0.05) (Fig. 2a). The effect of PD on the osteogenesis of hBMSCs was estimated by Alizarin red staining and qPCR. hBMSCs were cultured in OIM or OIM with PD for 21 days. As shown in Fig. 2b, PD, particularly at a concentration of 30 μM, increased calcium deposition at day 21, as shown by Alizarin red staining, which was consistent with the results of the Alizarin red staining (Fig. 2c). We further conducted qPCR to examine the expression of osteogenic marker genes (*OCN*, *RUNX2*, *β-catenin*, and *TAZ*) in hBMSCs induced with PD for 3 days. PD significantly promoted osteogenic gene expression in hBMSCs compared to that in cells treated with only OIM (Fig. 2d). In summary, 30 μM PD notably increased the proliferation and osteogenic differentiation of hBMSCs. Thus, this concentration was chosen for the following experiments.

**Fig. 2:** Polydatin promoted the proliferation and osteogenesis of hBMSCs. **a** PD with various concentrations notably stimulated hBMSCs to proliferate at 1, 2, 3, 7, and 14 days, particularly the 30 μM, according to the MTT assay results (*n* = 6). **b**, **c** hBMSCs were cultured in OIM with different concentrations PD (0, 10, 30, and 100 μM) for 21 days. The 30 μM PD significantly promoted the mineralization of hBMSCs (*n* = 3). **d** Following 3 days of PD treatments with various concentrations, *OCN*, *RUNX2*, *β-catenin*, and *TAZ* mRNA levels were measured by qPCR. *p < 0.05 versus the 0 μM group at the same time point, ^#^*p* < 0.05 versus the 10 μM group, and ^&^*p* < 0.05 versus the 30 μM group. OIM, osteogenic-induced medium. Results are shown as mean ± SD

### Effect of polydatin on the expression of osteogenic genes

We tested the effects of 30 μM PD on *TAZ*, *RUNX2*, *Osteopontin*, *DLX5*, *OCN*, *β-catenin*, *Collagen type I*, *BMP2*, and *OPG* expression during osteogenic differentiation of hBMSCs cultured in OIM at days 3, 7, and 14. The qPCR results showed that PD stimulation for 3, 7, and 14 days increased *TAZ*, *OCN*, *RUNX2*, *β-catenin*, *Collagen type I*, *BMP2*, and *OPG* mRNA levels (Fig. 3a, b, e–i), and PD stimulation for 3 and 7 days upregulated *Osteopontin* and *DLX5* mRNA levels (Fig. 3c, d).

**Fig. 3:** Polydatin (30 μM) increased *TAZ* (**a**), *RUNX2* (**b**), *Osteopotin* (**c**), *DLX5* (**d**), *OCN* (**e**), *β-catenin* (**f**), *Collagen type I* (**g**), *BMP2* (**h**), and *OPG* (**i**) expressions at the different stages of hBMSC osteogenesis. PD significantly stimulated the *RUNX2*, *Osteopotin*, *DLX5*, *β-catenin*, *Collagen type I*, and *BMP2* in the early period while TAZ, *OCN*, and *OPG* in later. Results are shown as the mean ± SD (*n* = 3). *p < 0.05, **p < 0.01, and ***p < 0.001 versus the PD group at the same time point, correspondingly

### Lentivirus-mediated TAZ shRNA offsets the effects of polydatin on osteogenic differentiation

Depletion of TAZ in hBMSCs was evaluated by using lentivirus-produced TAZ shRNA. The results of both qPCR and Western blot analysis showed that transfection with shTAZ2# significantly reduced the TAZ expression compared with that in the control and shCON-transfected groups (Fig. 4a, b). Moreover, shTAZ transfection blocked the PD-induced osteogenic differentiation of hBMSCs. This was supported by the results of the ALP activity assay and determination of the mRNA expression of osteogenic genes. The ALP activity was obviously decreased in the shTAZ+PD group compared with the shCON+PD group, and there were no significant differences in ALP activity among the shCON, shTAZ, and shTAZ+PD groups (Fig. 4c). Compared with the shCON+POL group, the shTAZ+POL group exhibited reduced mRNA expression of *RUNX2*, *Osteopontin*, *β-catenin*, and *DLX5* at day 3; *TAZ* expression at 7 days; and *OCN* expression at day 14 (Fig. 4d).

**Fig. 4:** TAZ knockdown offsets the polydatin-induced osteogenic differentiation of hBMSCs. **a** qPCR was used to test the knockdown efficiency of shTAZ (numbers 1, 2, and 3) at day 14. *p < 0.05 versus the control group; ^#^*p* < 0.05 versus the shCON group. **b** The expressions of TAZ protein in different groups were detected by Western blot at day 14. *p < 0.05 versus the control group; ^#^*p* < 0.05 versus the shCON group. **c** shTAZ transfection reduced the ALP activities of hBMSCs cultured in OIM with or without PD for 14 days. **d** shTAZ transfection markedly neutralizes the PD promotional effect on the expression of osteogenic genes (*n* = 3). *p < 0.05 versus the shCON group; ^#^*p* < 0.05 versus the shCON+POL group. POL, polydatin

### Polydatin increased total TAZ protein expression in hBMSCs mediated by the BMP2 and Wnt/β-catenin signaling pathways

Noggin and DKK1 are inhibitors of BMP2 and Wnt/β-catenin, respectively. Western blot analysis indicated that PD enhanced the expression of the TAZ protein on days 3 and 7 compared with that in the control group. However, this increase in expression induced by PD was blocked by Noggin and DKK1 (Fig. 5a, b). However, the change in p-TAZ Ser89 expression was contrary to that in TAZ expression; the level of p-TAZ Ser89 on days 3 and 14 was lower in the PD group than in the control group. However, the corresponding levels on days 3, 7, and 14 in the Noggin-treated groups were significantly higher than those in the PD group (Fig. 5c, d). In conclusion, our results showed that PD increased TAZ expression through the BMP2 and Wnt/β-catenin signaling pathways.

**Fig. 5:** Noggin and DKK1 countervail the PD promotion effect on the total TAZ protein, and Noggin further increases the expression of p-TAZ protein. hBMSCs were cultured in OIM with 30 μM PD for 3, 7, and 14 days, and the same amount of PBS was used in the control group. **a**, **b** Both Noggin and DKK1 attenuated the changes of TAZ protein in these time points. **c**, **d** However, DKK1 did not alter p-TAZ protein expression. Data are presented as mean ± SD (*n* = 3). *p < 0.05, **p < 0.01, and ***p < 0.001 versus the PD group at the same time point, correspondingly

### Polydatin-induced TAZ nuclear translocation in hBMSCs

To determine whether the effect of PD in activating hBMSC osteogenic differentiation was related to an increase in TAZ nuclear translocation, we conducted immunolabeling and fluorescence microscopy and found that 30 μM PD promoted the nuclear (blue) translocation of TAZ (red) in hBMSCs, which was hampered by Noggin and DKK1 (Fig. 6).

**Fig. 6:** PD promoted the nuclear translocation of TAZ in hBMSCs, but Noggin and DKK1 offset this effect. hBMSCs were cultured with OIM in the presence of PD, PD + Noggin, PD + DKK1, and the same amount of PBS as a control group for 7 days. TAZ with red fluorescence dyes and nuclei with blue were shown in these representative images

### PD inhibited estrogen deficiency-induced bone loss in OVX mice

To explore the effect of PD on estrogen deficiency-induced bone loss, OP model mice were treated with PD (3 mg/kg) or an equal volume DMSO alone as a control. The mice were sacrificed after 4, 8, or 12 weeks of treatment (Fig. 7a). The micro-CT scanning results revealed that PD significantly reduced ovariectomy-induced bone loss, as shown by the increased BV/TV, Tb.N, and Tb.Th in the OVX+PD group. Trabecular separation (Tb.Sp) was also decreased in the OVX+PD group compared with the OVX group (Fig. 7b, c). The H&E staining results also confirmed the improved trabecular structure in different groups after PD intervention (Fig. 8a). Immunohistochemistry proved that PD significantly stimulated the expression of TAZ and OPG in the bone (Fig. 8a, b). As shown by ELISA, PD suppressed the serum expression of the osteoclastic markers RANKL and β-CTX. The change in the expression of serum OPG was opposite that of the other two markers (Fig. 8c).

**Fig. 7:** PD inhibited OVX-induced bone loss in vivo. **a** Schematic images of the OVX mouse establishment and the experimental process to evaluate PD therapeutic effects. **b** Representative micro-CT images showed PD administration attenuated distal femoral bone loss. **c** Quantitative analyses of microstructure parameters, including bone volume per tissue volume (BV/TV), trabecular thickness (Tb.Th), trabecular separation (Tb.Sp), bone surface area per bone volume (BS/BV), structure model index (SMI), and trabecular number (Tb.N), *n* = 6 per group. Bars are shown as mean ± SD. *p < 0.05 versus the sham group; ^#^*p* < 0.05 versus the OVX+PD group

**Fig. 8:** PD improved the trabecular structure and stimulated the expression of the TAZ and OPG in OVX mice. **a** Representative images of HE and immunohistochemical staining of distal femoral trabecular bone. **b** Quantitative analyses of TAZ and OPG. **c** PD promoted the serum expression of OPG while inhibited RANKL and β-CTX. Data are presented as mean ± SEM. Scale bars, 100 μM. *p < 0.05 compare with the sham group, ^#^*p* < 0.05 versus the OVX+PD group

## Discussion

OP is a common bone disease characterized by low bone mass and subsequent elevated fracture risk [34]; therefore, antiresorptive agents, anabolic agents, and bone/mineral drugs have been used to maintain normal bone mass. However, their limitations and side effects, such as an increased risk of breast cancer, jaw necrosis, or atypical femur fracture, have gradually been found [35, 36]. Thus, the discovery of an alternative OP treatment with fewer side effects would be promising. Disordered proliferation and differentiation of BMSCs are the main causes of osteoporosis [37, 38], especially the impaired ability of BMSCs to differentiate into osteoblasts [39]. Therefore, the promotion of osteogenic differentiation can help inhibit the development of osteoporosis. According to the literature, herbal extracts, acting as stimulants of the proliferation and differentiation of hBMSCS, have outstanding effects, and their osteogenic, vascular, chondrogenic, and neurogenic potential should be further studied [40]. We therefore investigated the exact antiosteoporotic mechanism of a prominent Chinese compound, PD, in vitro and in vivo.

As described by our results, PD increased the proliferation and osteogenic differentiation of hBMSCs without cytotoxicity, as proven by the significant increases in calcium nodules and expression of osteoblast markers, which is consistent with the results of our previous study [31]. In our previous study, we also found that the PD-induced expression of BMP2 was not blocked by a specific Wnt signal inhibitor. Furthermore, it is illustrated that PD activated the BMP2-induced Wnt signaling pathway through enhancing the accumulation and nuclear translocation of β-catenin and subsequently promoted the osteogenesis of hBMSCs [31]. Further experiments found that knockdown of TAZ hampered the effect of PD on osteogenesis through the BMP2-Wnt/β-catenin signaling pathway. The increased bone mass of OVX mice also supported that the osteogenesis effect of PD is closely related to TAZ. Thus, we demonstrated that PD improves the osteogenic differentiation of hBMSCs by stimulating TAZ expression via the BMP2-Wnt/β-catenin signaling pathway.

The BMP and Wnt/β-catenin pathways engage in substantial crosstalk in preosteoblasts, and the Wnt pathway acts as a downstream regulator of BMPs to regulate the progression of proliferation, bone differentiation, and mineralization [41–43]. RUNX2 is the main regulatory factor that activates osteogenic differentiation through the BMP and Wnt/β-catenin signaling pathways. It can induce the nuclear translocation of β-catenin [44] and promote BMP2-induced osteogenic differentiation [45] and the binding of BMP2 with Wnt/β-catenin [16, 46]. Thus, the central mechanism of osteogenesis is executed by the BMP and Wnt signaling pathways [47]. More specifically, BMP2 stimulates bone formation through activating RUNX2 [48], and the Wnt/β-catenin pathway activates RUNX2 in MSCs through the transcriptional regulator TCF/LEF [49], while RUNX2 also promotes the expression of β-catenin [50].

Recently, TAZ was found to serve as a regulatory transcription coactivator for RUNX2-stimulated *OCN* gene expression and thus promote osteogenic differentiation of MSCs [51]. TAZ is widely known as a regulator of the Hippo pathway and a novel regulator of typical Wnt signaling [20, 52], but the specific mechanism by which TAZ promotes osteogenic differentiation has not been fully clarified. Azzolin et al. [53] found that Wnt can stabilize TAZ and β-catenin and stimulate their nuclear transfer, thus promoting osteoblastic differentiation. In addition, the presence of Wnt3a facilitates the interaction between TAZ and RUNX2, which significantly increases RUNX2-mediated osteogenic gene transcription [54]. Several studies have elaborated that TAZ stimulates the osteogenic differentiation of MSCs by increasing the expression of RUNX2 [22, 55, 56]. In addition, BMP2 not only increases TAZ expression but also promotes subsequent TAZ-stimulated expression of the OCN gene by RUNX2, which is essential for osteoblast differentiation [51]. Therefore, RUNX2 plays a vital role in the crosstalk between the BMP2 and Wnt/β-catenin pathways to regulate BMSC osteogenic differentiation, which is closely related to the interaction of RUNX2 with TAZ [57–60]. Consistent with these previous studies, we found that the knockdown of TAZ tremendously impeded the osteogenic effect of PD through the BMP2-Wnt/β-catenin pathway.

This hypothesis was confirmed by the increased bone mass of OVX mice after PD treatment. Remarkably, PD intervention significantly increased the expression of TAZ and OPG and decreased that of RANKL. The OPG/RANKL ratio plays a crucial role in OP. RANKL activates the receptor RANK to induce osteoclast differentiation, which is blocked by OPG, leading to the inhibition of osteoclast growth and bone resorption [61–63]. PD has been proven to alleviate the symptoms of OP in OVX mice by upregulating the expression of OPG and β-catenin and downregulating that of RANKL [30]. Combined with our in vitro results, these findings demonstrate that TAZ plays a key role in the process by which PD improves hBMSC osteogenic differentiation.

## Conclusion

In conclusion, PD could promote the proliferation and osteogenic differentiation of hBMSCs and maintain the bone matrix in an OVX mouse model through the regulation of BMP2 and the Wnt/β-catenin pathway, and TAZ plays a pivotal role in regulating this process (Fig. 9).

**Fig. 9:** Hypothetical scheme furtherly illustrates the mechanism of which polydatin improves osteogenic differentiation of hBMSCs via stimulating the expression of TAZ in the BMP2-Wnt/β-catenin pathway. And the interaction between Wnt-TAZ-RUNX2 can significantly stimulate the osteogenic differentiation

## Data Availability

The datasets used and/or analyzed during the current study are available from the corresponding author on reasonable request.

## Abbreviations

OP: Osteoporosis
ALP: Alkaline phosphatase
BMP2: Bone morphogenetic protein 2
DKK1: Dickkopf-related protein 1
DMSO: Dimethyl sulfoxide
OVX: Ovariectomized
PD/POL: Polydatin
hBMSCs: Human bone marrow stromal cells
OIM: Osteogenic induction medium
PBS: Phosphate-buffered saline
PFA: Paraformaldehyde PDZ-binding motif: TAZ
RUNX2: Runt-related transcription factor 2
DLX5: Distal-less homeobox 5
OPG: Osteoclastogenesis inhibitory factor
OCN: Osteocalcin
